This article has been retracted.

# The best drug supplement for obesity treatment: a systematic review and network meta-analysis

**DOI:** 10.1186/s13098-021-00733-5

**Published:** 2021-10-18

**Authors:** Nader Salari, Samira Jafari, Niloofar Darvishi, Elahe Valipour, Masoud Mohammadi, Kamran Mansouri, Shamarina Shohaimi

**Affiliations:** 1 Department of Biostatistics, School of Health, Kermanshah University of Medical Sciences, Kermanshah, Iran; 2 Student Research Committee, Kermanshah University of Medical Sciences, Kermanshah, Iran; 3 Zimagene Medical Genetics Laboratory, Avicenna St, Hamedan, Iran; 4 Department of Nursing, School of Nursing and Midwifery, Kermanshah University of Medical Sciences, Kermanshah, Iran; 5 Medical Biology Research Center, Kermanshah University of Medical Sciences, Kermanshah, Iran; 6 Department of Biology, Faculty of Science, University Putra Malaysia, Serdang, Selangor Malaysia

**Keywords:** Obesity, Treatment, Network-meta analysis

## Abstract

**Background:**

Obesity is a complex disease with an increasing prevalence worldwide. There are different weight-management options for obesity treatment, including dietary control, exercise, surgery, and medication. Medications are always associated with different responses from different people. More safety and efficacy of drugs with fewer side effects are valuable for any clinical condition. In this systematic review and network meta-analysis, different anti-obesity drugs are compared to identify the most effective drug.

**Methods:**

All relevant studies were extracted by searching national and international databases of SID, MagIran, ProQuest, PubMed, Science Direct, Scopus, Web of Science (WoS), and Google Scholar without time limit until October 2020. Finally, the meta-analysis was performed with the 11 remaining studies containing 14 different drug supplements. The standardized mean difference (SMD) was calculated at a 95% confidence interval (CI) to evaluate the effects of each treatment group compared with placebo. A random-effect model was used to evaluate the effect of individual studies on the final result. Heterogeneity and incompatibility of the network were assessed by Cochran’s Q and Higgins I^2^, and the Net Heat chart, respectively. Data analysis was performed using R software.

**Results:**

Our results showed that there were significant mean effects in people intervened with Phentermine 15.0 mg + Topiramate 92.0 mg, Phentermine 7.5 mg + Topiramate 46.0 mg, Pramlintide, Naltrexone + Bupropion 32, and Liraglutide, with SMD effects size = − 9.1, − 7.4, − 6.5, − 5.9, − 5.35, respectively.

**Conclusion:**

This study was performed to compare the effect of different drugs used for weight loss in obese patients. The most effective drugs for weight loss were phentermine and topiramate, pramlintide, naltrexone, bupropion, and liraglutide compared to placebo treatment, respectively. This study provides new insights into anti-obesity drugs and hopes to shed new light on future research to manage and treat obesity.

## Background

Today, obesity is a growing public health issue worldwide, with an increased risk for chronic and aggressive conditions such as respiratory complications, hypertension, diabetes mellitus, cardiovascular diseases, and cancer [1–3]. The increasing prevalence of overweight and obesity is seen in all age groups [2]. According to the WHO, in 2016, 39% of adults (≥ 18 years, 39% men, and 40% women) were overweight. According to the report, the global prevalence of obesity has almost tripled from 1975 to 2016.

With the impact of obesity on health, quality of life, and social function, its management interventions are of great value [4]. Different management approaches are used to control and treat obesity, which are determined based on age, sex, puberty status, the severity of obesity, underlying causes, obesity-related complications, psychosocial factors, and patient and family preferences [5]. Due to fewer side effects, behavioral and dietary modifications and more exercise are considered the first-line treatment for weight loss in obese patients [6, 7]. In addition, drug therapy is recommended for those whose lifestyle interventions alone are not responsive, especially if there is no possibility of bariatric surgery in these individuals [8]. The role of drugs in weight loss is controversial, and their effectiveness seems limited. It may be very effective for some people and not effective for others and may even have side effects for some [9, 10].

Phentermine is one of the oldest sympathomimetic drugs that contain diethylpropion. It is the most commonly used drug in the United States, accounting for 70% of prescriptions. The combination of phentermine and topiramate causes more weight loss than each of them separately [10]. Phentermine and topiramate extended-release (long-acting) capsules are used to help adults who are obese or who are overweight and have weight-related medical problems to lose weight and to keep from gaining back that weight [10].

Orlistat is a potent inhibitor of pancreatic lipase that reduces intestinal fat digestion [11]. Lorcaserin is a US food and drug administration (FDA)-approved selective agonist of the serotonin [5-hydroxytryptamine (5HT)]—2C receptor that is effective in weight loss by reducing appetite and increasing satiety [12]. This medication is used with a doctor-approved exercise, behavior change, and reduced-calorie diet program to help you lose weight, and taking orlistat can also help keep you from gaining back the weight you have lost [12].

Liraglutide, sold under the brand name Victoza, is an anti-diabetic medication used to treat type 2 diabetes, obesity, and chronic weight management [13]. Liraglutide is used as a supplement to low-calorie diets and increased physical activity to control chronic overweight in adults [13]. Naltrexone/bupropion (contrave) combines an opioid receptor antagonist (naltrexone) with a dopamine and norepinephrine reuptake inhibitor (bupropion) in an extended-release tablet; the combination of naltrexone and bupropion reduces hunger and does not affect energy metabolism [13].

Pramlintide is an injectable drug that lowers the glucose level in the blood, and it is used for treating type 1 and type 2 diabetes. Pramlintide is a synthetic hormone that resembles human amylin [11–13]. Lorcaserin, marketed under the brand name Belviq is a weight-loss drug developed by Arena Pharmaceuticals. It reduces appetite by activating a type of serotonin receptor known as the 5-HT2C receptor in a region of the brain called the hypothalamus, which is known to control appetite [11–13]. Several other drugs are used to treat obesity, but this systematic and network meta-analysis review focused on these mentioned drugs to determine which is the most effective drug in weight control [13].

Systematic reviews usually include a detailed and comprehensive plan that reduces bias to identify, evaluate, and integrate all studies on a particular topic [14]. This method is an essential tool for creating valid summaries of health care information for physicians and patients. Systematic reviews provide information on interventions' benefits and side effects and help develop clinical knowledge for future research [15].

In many clinical areas, physicians consider more than two alternative therapies, each of which may be compared to standard care, placebo, or alternative interventions. Due to the lack of direct or indirect comparison of some interventions with placebo, there may be challenges in selecting them and determining relative superiority. Network meta-analysis can help solve this problem so that in addition to providing useful information about interventions that no study has directly compared, it can increase the accuracy of estimating their impact by combining direct and indirect evidence [16]. For this reason, network meta-analysis is more powerful and accurate than binary meta-analysis.

There are three important hypotheses to perform a network meta-analysis: (1) similarity or transfer, different treatment studies need to be sufficiently similar in terms of clinical characteristics and methodology, including population and results; (2) Homogeneity in estimating the effect of experiments compared with similar treatments (i.e., having the same design); and (3) Compatibility in estimating the effect of different sources of evidence (from direct and indirect comparison) [17]. Incompatibility within the treatment network is assessed through the net heat diagram, a graphical tool in which blue indicates a low level of incompatibility, while red indicates "hot spots" of high incompatibility [18].

## Methods

This study was conducted through a systematic search of databases, organizing documents for review, selecting studies according to inclusion and exclusion criteria, extracting information, analyzing data, and presenting a final report based on Preferred Reporting Items for Systematic Reviews and Meta-Analyzes (PRISMA) [19].

### Inclusion and exclusion criteria

Inclusion criteria included: (1) RCT studies, (2) studies in English or Persian, and (3) studies of Pramlintide, Liraglutide, Lorcaserin, Naltrexone-Bupropion, Orlistat, Phentermine-topiramate used alone or in combination with other drugs mentioned in this list.

Exclusion criteria: (1) observational studies (case–control and cohort), (2) case report studies, Letter to editor (3) animal studies.

### Search strategy

For the systematic search of studies, national and international databases were examined. The two databases MagIran and SID from national databases were examined with Persian keywords. ProQuest, PubMed, Science Direct, Scopus, Web of Science (WoS), and Google Scholar search engines were examined with English keywords.

The keywords used to search in this study were selected from Medical Subject Headings (MESH Terms) after careful review of research questions and previous studies related to the title and based on PICO criteria (Participants: obese or overweight people; Intervention: based on treatment with Pramlintide, Liraglutide, Lorcaserin, Naltrexone-Bupropion, Orlistat, Phentermine-topiramate; Comparison: between the effects of the mentioned drugs on weight loss in participants; Outcomes: determining the most effective drug in weight loss that is considered as a result of the study [20]). Selected keywords including obesity, pharmacological treatment, appetite control, and synonyms were combined with the Boolean search method. The references of the studies were also reviewed to find more relevant empirical studies.

### Information extraction and quality evaluation

After extracting the data, the treatments were grouped into 14 classes including Pramlintide, Liraglutide, Liraglutide 1.8, Liraglutide 0.3, Lorcaserin, Lorcaserin QD, Lorcaserin BID, Naltrexone-Bupropion, Orlistat QD, Orlistat BID, Phentermine 15.0 mg + Topiramate 92.0 mg, Phentermine 7.5 mg + Topiramate 46.0 mg, Naltrexone + Bupropion 32, Naltrexone + Bupropion 16.

Mean and standard deviation before and after treatment were extracted for both case and control groups to calculate the effect size as the standardized mean difference (SMD). In the absence of the mean and standard deviation after treatment, mean and standard deviation were calculated using mean weight and standard deviation before treatment, respectively. In studies with different mean changes, absolute change was considered. The last week of the course of the desired drug treatment was considered to extract information. In studies with unknown communities of Intention-to-treat (ITT) and Completers, data were extracted according to the evidence. Also, studies with unknown populations were considered as Intention-to-treat (ITT) populations.

For qualitative evaluation, validation, and critique of intervention studies, the CONSORT checklist is usually used [21], which consists of six general sections, including title, abstract, introduction, methods, results, and discussion. Some of these sections have subsections, and in total, a manuscript contains 37 items. These 37 items include various aspects of the study methodology, including title, problem statement, study objectives, study type, statistical study population, sampling method, determining the appropriate sample size, defining variables and procedures, study data collection tools, statistical analysis methods, and findings. Accordingly, the maximum score obtained from the qualitative evaluation in the CONSORT checklist will be 37. Therefore, considering a score of 17 as the cut-off point, studies with a score of ≥ 17 were considered good and average methodological quality, and studies with a score of < 17 were considered poor methodological quality, so they were excluded from the study.

### Statistical analysis

The SMD effect size was estimated for the differences of the groups due to the change from the beginning. In each study, data from participants who performed post-treatment assessments were used. Network meta-analysis calculations were performed using statistical software package R 3.6.3, and frequency-oriented network meta-analysis was performed using the Net-meta package. Cochran’s Q and Higgins I^2^ were calculated to investigate the network heterogeneity. Cochran’s Q is calculated as a weighted sum of squares of the differences between the effects of a single study and the effect accumulated throughout the studies. Significant values indicate a high level of heterogeneity that needs to be further investigated [22]. Higgins I^2^ evaluates the variability in effect estimation resulted from heterogeneity between studies rather than chance. Low percentages indicate low heterogeneity, while percentages above 75% indicate a significant level of heterogeneity [23].

To evaluate the geometry of the network, the Net-graph function of the Net-meta package was used. In addition, pure net heat was used to detect hot spots of incompatibility in comparisons. The share of direct evidence merged from each individual plot (columns) in each grid estimate (rows) is shown with an area of gray squares. The colors in the diagram indicate the severity of the network incompatibility, the red squares (hotspots) indicate more incompatibility, and the blue squares indicate less incompatibility [24].

A trial and error method was performed by excluding a group of studies, depending on the possible confounding variables to explore the source of heterogeneity. Possible sources of variance calculated in the network included the average age of individuals, sample size, gender, negative values of effect size, year of publication of articles.

## Results

According to PRISMA guidelines, studies conducted in the field of drug treatment for obesity were systematically reviewed. Based on the initial search in the reviewed databases, 1456 studies were collected and transferred to the information management software (EndNote). Of these, 130 were repeated studies, 522 were unrelated, and 793 were excluded by reviewing the title and abstract based on inclusion and exclusion criteria. After evaluating the full text of the remaining 11 studies, all of these studies received good methodological quality based on the score obtained from the CONSORT checklist. After the quality assessment, these 11 studies entered the final analysis (Fig. 1). Information on these 11 studies is given in Table 1.

**Fig. 1:** The flowchart indicating the steps involved in reviewing the studies included in the systematic review and meta-analysis (PRISMA 2009)

**Table 1:** Information of studies included in the analysis step. mean age, sex and supplement type

Row	First author	Publication year	Setting	Mean age		Total patients	Supplement type	Men/women
				Intervention	Control			
1	Apovian [25]	2013	America	44.3 ± 11.2	44.4 ± 11.4	1496	Placebo	76/419
							Naltrexone + bupropion	155/846
2	Aronne [26]	2010	America	42 ± 11	42 ± 11	244	Placebo	13/87
							Pramlintide	12/88
3	Davies [27]	2015	France, Germany, Israel, South Africa, Spain, Sweden, Turkey, United Kingdom		57.4 ± 9.8	864	Placebo	97/115
							Liraglutide 0.3 mg	220/203
							Liraglutide 1.8 mg	108/103
4	Fidler [28]	2011	America	BID: 43.8 ± 11.8	43.7 ± 11.8	4004	Placebo	353/1248
				QD: 43.8 ± 11.7			Lorcaserin 10 mg BID	313/1289
							Lorcaserin 10 mg QD	145/656
5	Gadde [29]	2011	America	(7.5 mg + 46 mg): 51.1 ± 10.43	51.2 ± 10.25	2487	Placebo	299/695
				(15 mg + 92 mg): 51.0 ± 10.65			Phentermine 7.5 mg + topiramate 46.0 mg	149/349
							Phentermine 15.0 mg + topiramate 92.0 mg	302/693
6	Greenway [30]	2010	America	16 mg: 44.4 ± 11.3	43.7 ± 11.1	1742	Placebo	85/496
				32 mg: 44.4 ± 11.1			Naltrexone + bupropion 16.0 mg	88/490
							Naltrexone + bupropion 32.0 mg	87/496
7	le Roux [31]	2017	America	47.5 ± 11.7	47.3 ± 11.8	2254	Placebo	176/573
							Liraglutide	364/1141
8	Lu [32]	2018	China	34.7 ± 9.0	37.0 ± 10.0	171	Placebo	28/57
							Lorcaserin	39/46
9	O’neil [33]	2012	America	BID: 53.9 ± 8.1	53.2 ± 8.3	508	Placebo	73/84
				QD: 53.5 ± 7.4			Orlistat 120.0 mg BID	86/83
							Orlistat 120.0 mg QD	34/41
10	Pi-Sunyer [34]	2015	Europe, North America, South America, Asia, Africa, Australia	45.0 ± 12.0	45.2 ± 12.1	3731	Placebo	273/971
							Liraglutide	530/1957
11	Smith [35]	2010	America	43.8 ± 0.3	44.4 ± 0.3	3182	Placebo	253/1331
							Lorcaserin	272/1321

In the study by Apovian et al., which evaluated the effect of Naltrexone + Bupropion and Placebo; weight change was reduced by 7.9 ± 0.3 and 1.5 ± 0.5, respectively [25]. Aronne et al.’s study of the effects of Pramlintide and placebo showed a weight change of 3.6 ± 0.7 and 2.1 ± 0.9, respectively [26]. The study by Davies et al. also reported weight changes of 5, 6.4, and 2.2, respectively, in the effect of Liraglutide 1.8 mg, Liraglutide 0.3 mg, and placebo [27]. In the results presented in Table 2, weight change as a result of taking Lorcaserin 10 mg BID, Lorcaserin 10 mg QD, and placebo were 5.8, 4.7, and 2.9, respectively [28] (Table 2).

**Table 2:** Information of studies included in the analysis step. Initial mean weight (kg), Mean weight change (kg) and Final mean weight (kg)

Row	First author	Publication year	Supplement type	Initial mean weight (kg)	Mean weight change (kg)	Final mean weight (kg)	P-value
1	Apovian [25]	2013	Placebo	99.2 ± 15.9	− 1.5 ± 0.5	97.7 ± 15	< 0.001
			Naltrexone + bupropion	100.3 ± 16.6	− 7.9 ± 0.3	92.4 ± 11	
2	Aronne [26]	2010	Placebo	107 ± 22	− 2.1 ± 0.9	104.9 ± 21	< 0.05
			Pramlintide	102 ± 19	− 3.6 ± 0.7	98.4 ± 18.5	
3	Davies [27]	2015	Placebo	106.5 ± 21.3	− 2.2	104.3 ± 20	< 0.001
			Liraglutide 0.3 mg	105.7 ± 21.9	− 6.4	99.3 ± 18.9	
			Liraglutide 1.8 mg	105.8 ± 21	− 5	100.8 ± 19	
4	Fidler [28]	2011	Placebo	100.8 ± 16.2	− 2.9 ± 6.4	97.9 ± 15	< 0.001
			Lorcaserin 10 mg BID	100.3 ± 15.7	− 5.8 ± 6.4	94.5 ± 12	
			Lorcaserin 10 mg QD	100.1 ± 16.7	− 4.7 ± 6.4	95.4 ± 13.5	
5	Gadde [29]	2011	Placebo	103.3 ± 18.1	− 1.4	101.9 ± 17.5	< 0.0001
			Phentermine 7.5 mg + topiramate 46.0 mg	102.6 ± 18.2	− 8.1	94.5 ± 15.5	
			Phentermine 15.0 mg + topiramate 92.0 mg	103 ± 17.6	− 10.2	92.8 ± 10.6	
6	Greenway [30]	2010	Placebo	99.5 ± 14.3	− 1.9 ± 0.5	97.6 ± 14	< 0.0001
			Naltrexone + bupropion 16.0 mg	99.5 ± 14.8	− 6.5 ± 0.5	93 ± 11.5	
			Naltrexone + bupropion 32.0 mg	99.7 ± 15.9	− 8 ± 0.5	91.7 ± 12	
7	le Roux [31]	2017	Placebo	107.9 ± 21.8	− 2 ± 7.3	105.9 ± 21	< 0.0001
			Liraglutide	107.5 ± 21.6	− 6.5 ± 8.1	101 ± 18	
8	Lu [32]	2018	Placebo	91.5 ± 14.5	− 3.6	87.9 ± 13	0.044
			Lorcaserin	92.6 ± 13.3	− 5.8	86.8 ± 10	
9	O’neil [33]	2012	Placebo	101.6 ± 18.1		101.7 ± 18.3	
			Orlistat 120.0 mg BID	104.7 ± 17.9		104.7 ± 17.9	
			Orlistat 120.0 mg QD	105.9 ± 19.0		105.4 ± 19.2	
10	Pi-Sunyer [34]	2015	Placebo	106.2 ± 21.7	− 2.8 ± 6.5	103.4 ± 20	< 0.001
			Liraglutide	106.2 ± 21.2	− 8.4 ± 7.3	97.8 ± 17	
11	Smith [35]	2010	Placebo	99.7 ± 0.4	− 2.2 ± 0.1	97.5 ± 0.4	< 0.001
			Lorcaserin	100.4 ± 0.4	− 5.8 ± 0.2	94.6 ± 0.4	

### Network meta-analysis results

At the beginning of the study, 36 studies were extracted, and their effect size (TE) and standard error (seTE) values were calculated with the appropriate instructions. The relevant studies and values were stored in a separate Excel file and entered in the analysis step. Of these 36 studies, one study included five arms, seven studies included three- arms, and the rest included two arms.

After performing a network meta-analysis with these studies, a single network was not formed, but seven sub-networks were obtained (Q = 3743.17 and I^2^ = 99.6%). High values of I^2^ and Q indicated high heterogeneity and incompatibility of the studies. Studies with a common placebo (26 studies) were separated, and instructions were executed for them to solve this problem. One study was then excluded due to high incompatibility (Erondu, N). By re-executing the instructions, a single network was formed but with high values of I^2^ and Q (Q = 1177.94 and I^2^ = 98.6%).

In order to achieve greater homogeneity, the commonality of the intervention was considered in addition to placebo. Therefore, 19 studies were selected from these 26 studies. There were four treatments at this stage: Placebo, Liraglutide, Orlistat, and Lorcaserin. But I^2^ and Q had high values (Q = 1177.94 and I^2^ = 98.6%) after executing instructions. Studies related to Lorcaserin were excluded due to few numbers. Seventeen studies remained after executing the instructions, high values were obtained for I^2^ and Q (Q = 1176.92 and I^2^ = 98.7%).

Finally, the column indicating effect size (TE) was sorted from small to large, and the first five studies were considered. After executing the instructions, a significant decrease was observed in the values of I^2^ and Q (Q = 3.32 and I^2^ = 9.6%). Thus, a small network with five studies and with high homogeneity was formed. Subsequently, five other studies were added to the small network, and instructions were executed. If a sub-network was formed, the first binary groups of studies are considered. If the sub-network was formed again, the studies are considered one by one to find the heterogeneity factor. According to this method, eventually, a large network was formed with 28 desired studies. Q and I^2^ values for this network were 1194.92 and 98.5%, respectively, which are high values. The network diagram is also shown in Fig. 2. The graph of net heat is shown in Fig. 3. Due to the high degree of heterogeneity, analysis of the random-effect model seems to be more appropriate. The net heat diagram shown in Fig. 4 indicates a significant decrease in incompatibility.

**Fig. 2:** The network diagram obtained from the preliminary results of a review of various drug supplements used in the treatment of obesity in the worldwide

**Fig. 3:** The graph of net heat obtained from the preliminary results of a review of various drug supplements used in the treatment of obesity in the worldwide

**Fig. 4:** The net heat diagram obtained from the final results of a review of various drug supplements used in the treatment of obesity in the worldwide, based on the random-effect model after removing heterogeneous items

Other characteristics examined in the studies can also be considered to achieve greater homogeneity. For example, considering the mean age of individuals and exclusion of studies with different mean ages, no change was observed in the values of I^2^ and Q (Q = 1171.14 and I^2^ = 98.7%). Here, two studies with mean ages of 14.4 and 13.5 were excluded [36], 37. Nevertheless, due to a slight change in I^2^ and Q, these studies were returned to the study.

In addition, the exclusion of studies with a sample size < 100 was examined. Three studies were excluded; Ariel, D [38], Halawi, Houssam [39], and Danne, Thomas [36]. According to the values of I^2^ and Q (Q = 1049.19 and I^2^ = 98.6%), these three studies were also restored to the study.

The sample size in women and men can also be considered. Here, the number of women was more than men in all studies. The studies can be re-reviewed by determining the conditions that create a high difference. For example, after exclusion studies with ratios of the number of women to the number of men more than five (seven studies were excluded; Finer, N [40], Apovian, CM [25], Greenway, Frank L. [30], Smith, Steven R [35], Rössner, Stephan [41], Davidson, Michael H [42] and Krempf, M [43]), The value of Q decreased, but the value of I^2^ was still high (Q = 798.03 and I^2^ = 98.9%), so the articles were returned to the study.

Furthermore, considering the mean weights before and after the intervention and the exclusion of studies with negative effect size (Davies, Melanie J [27], Fidler, Meredith C [28] and O’neil, Patrick M [33]), high values for I^2^ and Q obtained (Q = 1042.39 and I^2^ = 98.7%), and therefore these studies were returned to the study.

Moreover, based on the year of publication and exclusion studies published before 2010, I^2^ and Q values significantly reduced and balanced (Q = 8.22 and I^2^ = 63.5%). So these 14 studies were excluded from the study (Finer, N [40], Hanefeld, M [44], Bakris, George [45], Chanoine, JP [37], Swinburn, Boyd A [46], Sjöström, Lars [47], Rössner, Stephan [41], Broom, I [48], Davidson, Michael H [42], Hauptman, Jonathan [49], Kelley, David E [50], Krempf, M [43], Lindgärde, F obot [51], Miles, John M [52]). Finally, the network was formed with the remaining 11 studies (Fig. 5).

**Fig. 5:** The final network diagram obtained from the final results of the review of various drug supplements used in the treatment of obesity in the worldwide after removing heterogeneous items

According to the final network diagram, 21 pairwise comparisons were made. Comparing each treatment group with placebo indicated that there was significant mean effect in patients receiving Phentermine 15.0 mg + topiramate 92.0 mg, Phentermine 7.5 mg + topiramate 46.0 mg, Pramlintide, altrexone + bupropion 32, Liraglutide, with SMDs − 9.1 [CI 95% (− 7.826, − 10.374)], − 7.4 [CI 95% (− 5.6556, − 9.1444)], − 6.5 [CI 95% (− 13.4579, 0.4579)], − 5.9 [CI 95% (− 7.3896, − 4.4104)], − 5.35 [CI 95% (− 6.3983, − 4.3121)], respectively (Fig. 6).

**Fig. 6:** Meta-analysis study of various drug supplements used in the treatment of obesity in the worldwide based on a random-effect model

## Discussion

The purpose of this systematic review and network meta-analysis was to combine studies related to the effects of different drugs used for obesity treatment and to identify the most effective drugs for weight loss in obese people. There was high heterogeneity between studies, and this had a significant influence on the results. Numerous sources of heterogeneity were considered. After the trial and error method, the year of publication of studies was considered the most important and effective source of heterogeneity. Accordingly, studies published before 2010 were excluded. The network was formed with 11 studies. Drug including Pramlintide, Liraglutide, Liraglutide 1.8, Liraglutide 0.3, Lorcaserin, Lorcaserin QD, Lorcaserin BID, Naltrexone-Bupropion, Orlistat QD, Orlistat BID, Phentermine 15.0 mg + Topiramate 92.0 mg, Phentermine 7.5 mg + Topiramate 46.0 mg, Naltrexone + Bupropion 32, and Naltrexone + Bupropion 16 were compared with Placebo group.

Eating less and moving more are the basics of weight loss that lasts. For some people, prescription weight loss drugs may help. You will still need to focus on diet and exercise while taking these drugs, and they are not for everyone [53–55].

Doctors usually prescribe them only if BMI is 30 or higher, or if it is at least 27, and people have a condition that may be related to the weight, like type 2 diabetes or high blood pressure. When this action is combined with behavior changes, including healthy eating and increased physical activity, prescription medications help some people lose weight and maintain weight loss [55–57]. On average, after one year, people who take prescription medications as part of a lifestyle program lose 3% to 12% more of their starting body weight than people in a lifestyle program who do not take medication [53–57].

Research shows that some people taking prescription weight management medications lose 10% or more of their starting weight [51–57], weight loss of 5–10% of starting body weight may help improve health by lowering blood sugar, blood pressure and triglyceride levels. Losing weight also can improve some other health problems related to overweight and obesity, such as joint pain and sleep apnea. Possible side effects vary by medication and how it acts on your body. Most side effects are mild and often improve if you continue to take the medication [51–55].

How long you will need to take weight management medication depends on whether the drug helps you lose weight and keep it off and whether you experience serious side effects [53–57].

The key message for patients with obesity is that when caloric intake is reduced below that needed for daily energy expenditure, there is a predictable rate of weight loss. Men generally lose weight slightly faster than women of similar height and weight on any given diet because men have more lean body mass and, therefore, higher energy expenditure [58–61].

Available medications to help treat the patient with obesity work either in the brain or the gut. Neurotransmitter systems are involved in modulating food intake. Serotonin 5-HT2C receptors modulate fat and caloric intake [58–61].

α1-receptor agonist drugs used to treat hypertension produce weight gain. In contrast, stimulation of α2-receptors increases food intake, and a polymorphism in the α2a-adrenoceptor is associated with reduced metabolic rate in humans. Activation of β2-receptors in the brain reduces food intake, and β-blocker drugs can increase body weight. Other drugs act in the periphery; Glucagon-like peptide-1 released from intestinal L cells acts on the pancreas and brain to reduce food intake. Amylin is secreted from the pancreas and can reduce food intake [58–61].

A study by Smith et al. introduced the combination weight-loss drug Phentermine + Topiramate as a dietary supplement to manage the weight of obese or overweight patients and weight-related diseases [53].

There was also a significant mean efficacy for Pramlintide treatment compared with placebo. Pramlintide is an analogue of human amylin, FDA approved and used along with insulin in patients with type 1 and 2 diabetes. In addition to regulating glucose, Pramylintide increases satiety and thus reduces calorie intake through the central mechanism. It also facilitates moderate weight loss in obese or overweight patients with and without diabetes [54].

The combination drug Naltrexone and Bupropion also showed greater effectiveness in weight loss compared to placebo treatment. This combination drug is a weight control agent in Europe and a dietary supplement with reduced calories and increased physical activity in obese and overweight adults. In four randomized clinical trials, participants receiving this combination drug showed a weight loss of approximately three to five times that of those receiving placebo [55].

The result that Liraglutide helps reduce weight in obese patients was consistent with a study by Mehta et al. Liraglutide is effective in weight loss and its maintenance in obese patients, including patients with hypertension, dyslipidemia, type 2 diabetes, and obstructive sleep apnea. Comparative data in this study showed that weight loss with Liraglutide is more than drugs such as Orlistat or Lorcaserin [56].

A meta-analysis study by Khera et al. examined 28 randomized clinical trials with 29,018 obese and overweight patients to find a link between obesity drug treatments, weight loss, and side effects. Similar to the present study, they compared the drugs Orlistat, Lorcaserin, Naltrexone-Bupropion, Phentermine-Topiramate, and Liraglutide with another active ingredient or placebo in overweight or obese adults. Finally, it was reported that each of these drug treatments was associated with at least 5% weight loss at 52 weeks. And according to the estimated odds ratio values, Phentermine-Topiramate and Liraglutide were recognized as the most effective drugs [58].

In a randomized, double-blind, placebo-controlled trial, Danne et al. examined Liraglutide’s safety, tolerability, and pharmacokinetics in adolescents with obesity. In their study, 22 obese individuals were assigned in two groups to receive Liraglutide and placebo randomly and concluded that Liraglutide administration in obese adolescents had similar safety and tolerability characteristics to adult administration. No unexpected safety/tolerance issues were observed, and similar to the present study results, it can be said that Liraglutide is a suitable drug for adolescent weight loss [36].

Aronne et al. evaluated Phentermine and Topiramate compared to a combination of these drugs in a 28-week. Consistent with our results, they concluded that the combination of these drugs produced more weight loss than when each was used as a separate treatment [26].

The efficacy and safety of Naltrexone and Bupropion for obesity treatment were evaluated in a study by Georgios A. Christou and Dimitrios N. Kiortsis. Consistent with our results, they reported that this combination drug is an effective supplement for achieving weight loss and treating obesity-related diseases.

The small number of studies for some treatment methods was a limitation of this study that could affect the results. Also, due to the heterogeneity and inconsistency in the initial studies, many studies were excluded. In this study, the exclusion of studies published before 2010 had a significant impact on the homogeneity of results. Nevertheless, it is suggested that these excluded studies be covered in future meta-analyses.

## Conclusion

Different studies have been used to evaluate the effectiveness of drugs in the treatment of obesity. However, the results of these studies are different for different drugs and have heterogeneous results. The present study used a network meta-analysis to obtain the best supplements and drugs and provided the physician with the statistical and visual significance of the effect of each drug for treatment measures, and patients can also identify effective drugs. This study was performed to compare the effect of different drugs used in reducing the average weight of obese patients. The most effective drugs for weight loss were phentermine and topiramate, pramlintide, naltrexone, bupropion, and liraglutide compared to placebo treatment, respectively.

## Data Availability

Datasets are available through the corresponding author upon reasonable request.

## Abbreviations

SMD: The standardized mean difference
CI: Confidence interval
FDA: Food and drug administration
MESH: Medical subject headings
CONSORT: Consolidated standards of reporting trials
ITT: Intention-to-treat
NMA: Network meta-analysis
WoS: Web of Science
SID: Scientific information database
PRISMA: Preferred reporting items for systematic reviews and meta-analysis
